The article "Prognostic roles of the transcriptional expression of exportins in hepatocellular carcinoma" was published in 2019. Journal: Biosci Rep.

# Prognostic roles of the transcriptional expression of exportins in hepatocellular carcinoma

**DOI:** 10.1042/BSR20190827

**Published:** 2019-08-19

**Authors:** Lubiao Chen, Yanlin Huang, Liang Zhou, Yifan Lian, Jialiang Wang, Dongmei Chen, Huan Wei, Mingsheng Huang, Yuehua Huang

**Affiliations:** 1 Department of Infectious Diseases, The Third Affiliated Hospital of Sun Yat-sen University, Guangzhou, China; 2 Department of Interventional Radiology, The Third Affiliated Hospital of Sun Yat-sen University, Guangzhou, China; 3 Department of Critical Care Medicine, The First Affiliated Hospital of Guangzhou Medical University, Guangzhou, China; 4 Guangdong Provincial Key Laboratory of Liver Disease Research, The Third Affiliated Hospital of Sun Yat-sen University, Guangzhou, China

**Keywords:** Exportin, GEPIA, Hepatocellular carcinoma, ONCOMINE, Prognosis

## Abstract

**Aims:** A large number of studies have suggested that exportins (XPOs) play a pivotal role in human cancers. In the present study, we analyzed XPO mRNA expression in cancer tissues and explored their prognostic value in hepatocellular carcinoma (HCC).

**Methods:** Transcriptional and survival data related to XPO expression in HCC patients were obtained through the ONCOMINE and UALCAN databases. Survival analysis plots were drawn with Gene Expression Profiling Interactive Analysis (GEPIA). Sequence alteration data for XPOs were obtained from The Cancer Genome Atlas (TCGA) database and c-BioPortal. Gene functional enrichment analyses were performed with Database for Annotation, Visualization and Integrated Discovery (DAVID).

**Results:** Compared with normal liver tissues, significant XPO mRNA overexpression was observed in HCC cancer tissues. There was a trend of higher XPO expression in more advanced clinical stages and lower differentiated pathological grades of HCC. In HCC patients, high expression of XPO1, CSE1L, XPOT, XPO4/5/6 was related to poor overall survival (OS), and XPO1, CSE1L and XPO5/6 were correlated with poor disease-free survival (DFS). The main genetic alterations in XPOs involved mRNA up-regulation, DNA amplification and deletion. General XPO mutations were remarkably associated with worse OS and mostly affected the pathways of RNA transport and oocyte meiosis.

**Conclusion:** High expression of XPOs was associated with a poor prognosis in HCC patients. XPOs may be exploited as good prognostic biomarkers for survival in HCC patients.

## Introduction

Hepatocellular carcinoma (HCC) was the sixth most frequently diagnosed cancer and the fourth leading cause of cancer-related deaths worldwide in 2018, with almost 841000 new cases and 782000 deaths annually [1]. Although treatments including surgical resection, liver transplantation, radiofrequency or microwave ablation, transarterial chemoembolization and tyrosine kinase inhibitors (sorafenib, lenvatinib etc.) have been applied, the 5-year overall survival (OS) of HCC patients has not significantly improved [2]. The high mortality of HCC may be attributed to a delayed diagnosis and highly malignant biological behavior, including remote or intrahepatic metastasis, portal vein cancer thrombosis and intrahepatic bile duct obstruction [3,4]. A large number of investigations have explored the development and progression of HCC. However, to date, the molecular characteristics of HCC remain elusive. Identifying tumor pathogenesis in HCC is pivotal for revealing the mechanisms of hepatocarcinogenesis and will be helpful in developing effective therapies.

The trafficking of macromolecules through the nuclear envelope is essential for signal transduction and the regulation of a multitude of biological pathways. Defective nuclear transport may lead to changes in the physiological levels and space-time location of tumor suppressor genes and oncogenes, which might be ultimately associated with cellular differentiation and tumorigenesis [5–7]. The genes that undertake the tasks of shuttling cargo proteins from the cytoplasm into the nucleus by β-importins and from the nucleus out to the cytoplasm by exportins have been identified as those in the karyopherin-β family [8,9]. An overall study on different karyopherin-β family members in HCC would help reveal the molecular mechanism of the occurrence and development of HCC and provide insight into a new prognostic and therapeutic target for this deadly disease.

To date, seven exportins (XPOs) have been identified in humans and are encoded by XPO genes [10]. All of them take part in the transport of proteins/peptides and DNAs/RNAs from the nucleus out to the cytoplasm [7]. These exportins share common characteristics, with similar molecular weights (95–145 kDa), acid isoelectric points (4.0–5.5), low sequence identity (<20%) and helical HEAT repeats [11]. Previous studies have found the aberrant expression and prognostic values of some members of the XPO family in various cancers. For instance, XPO1 was identified as a key gene that plays a critical role in HCC by dynamic transcriptome analysis [12]. Consistent with these results, Zheng et al. [13] reported that XPO1 was overexpressed in HCC tissues compared with normal liver tissue. XPOT (also named as XPO3) was up-regulated in HCC tissues, and its overexpression was associated with poor OS. Further evidence suggested that XPOT might affect tumor progression via the cell cycle and ubiquitin-mediated proteolysis [14]. In contrast, Liang et al. found that the mRNA levels of XPO4 were down-regulated in liver cancerous tissues compared with paracancerous tissues, and this down-regulation predicted a poor prognosis [15,16]. Correspondingly, Li et al. [17] reported that XPO5 functioned as a cancer suppressor in the development and progression of HCC. Therefore, the roles of distinct XPO family members in HCC need to be further clarified.

In the present study, we addressed these issues by analyzing the expression of and mutations in different XPO members in patients with HCC. We also investigated the predictive functions of mutations in XPOs. Our results suggested that XPO family members have a significant impact on HCC progression. Therefore, XPOs could be used as potential biomarkers for predicting prognosis in HCC patients.

## Materials and methods

### ONCOMINE database analysis

The online cancer microarray database (ONCOMINE, http://www.oncomine.org) for gene expression was utilized in the present study. Data regarding the transcriptional mRNA expression of XPOs between HCC cancer samples and corresponding normal liver samples were obtained from this database. The differences were compared by using Student’s *t* test, and the statistical analysis parameters were set as follows: *P*-value <0.05, fold change = 1.5, gene rank = 10% and data type is mRNA [18].

### UALCAN analysis

UALCAN (http://ualcan.path.uab.edu) is an interactive web source based on level 3 RNA-seq and clinical data from 31 cancer types in The Cancer Genome Atlas (TCGA) database. UALCAN provides web resources for cancer researchers and clinicians to analyze the relative expression of potential genes in cancer and normal samples, to obtain the relative clinicopathological parameters, to draw survival analysis plotters, to estimate the impact of gene expression level and clinicopathological parameters on patient survival, and to identify novel genes in various individual cancer types [19]. Differences in transcriptional expression were compared by Student’s *t* test and a *P*-value <0.05 was considered statistically significant. The expression level was normalized as transcripts per million (TPM) reads for comparison across groups and individuals.

### Gene Expression Profiling Interactive Analysis

Gene Expression Profiling Interactive Analysis (GEPIA, http://gepia.cancer-pku.cn), an online cancer microarray database, was used to analyze the impact of the XPO family on the OS and disease-free survival (DFS) of HCC patients. Patients were divided into high expression and low expression groups according to the median expression level and assessed by Kaplan–Meier curves [20]. A *P*-value <0.05 was considered statistically significant.

### TCGA database analysis

TCGA (https://cancergenome.nih.gov/), a comprehensive and coordinated project aiming at improving diagnosis methods, treatment criteria and ultimately preventing cancer, had been assisting users to analyze large groups of over 30 human tumors through its genome analysis technologies, including large-scale genome sequencing and pathological data analysis [21].

### c-BioPortal database analysis

c-BioPortal (www.cbioportal.org) is an online open access resource for exploring, visualizing and analyzing multidimensional cancer genomics data. In the present study, c-BioPortal was used to access Liver Hepatocellular Carcinoma (TCGA, Provisional) data. The selected genomic profiles contained mutations, putative copy number alterations from GISTIC and mRNA expression z-Scores (RNASeq V2 RSEM). Seven target XPO family members were automatically calculated using a Z-score ±2.0. OncoPrint, OS or DFS plotter were obtained according to the online instructions at c-BioPortal [22].

### Gene Ontology and Kyoto Encyclopedia of Genes and Genomes pathway enrichment analyses

The Database for Annotation, Visualization and Integrated Discovery (DAVID, https://david.ncifcrf.gov/) was used to perform Gene Ontology (GO) and Kyoto Encyclopedia of Genes and Genomes (KEGG) analyses of all seven XPO genes. The human genome was selected as the background parameter. A *P*-value <0.05 was set as the threshold to indicate a statistically significant difference [23].

## Results

### High transcriptional expression of XPOs in HCC

To explore the expression of XPOs in HCC cancer tissue, the ONCOMINE and UALCAN databases were used to analyze their mRNA levels. As shown in Figure 1 and Table 1, compared with normal liver tissues, XPO1 mRNA levels exhibited a 1.642-fold (Roessler liver dataset [24], *P*=2.27e-09), 1.683-fold (Roessler liver 2 dataset [24], *P*=9.79e-54) and 1.782-fold (Wurmbach liver dataset [25], *P*=2.65e-07) increase in HCC cancer tissues. CSE1L (also named as XPO2) was also found to be 2.209-fold (Roessler liver dataset [24], *P*=2.02e-08), 2.218-fold (Roessler liver 2 dataset [24], *P*=2.77e-75) and 1.914-fold (Wurmbach liver dataset [25], *P*=2.16e-05) increased in HCC cancer tissues. In contrast, a −2.482-fold decrease in CSE1L mRNA levels was found in another HCC study (Chen Liver dataset [26], *P*=4.27e-06). Likewise, XPOT mRNA levels increased 2.245-fold (Roessler liver dataset [24], *P*=8.41e-63) and 1.763-fold (Chen liver dataset [26], *P*=4.01e-14) but decreased −2.122-fold in HCC cancer tissues in another HCC dataset (Mas liver dataset [27], *P*=4.32e-07). Similarly, the XPO5 mRNA level was increased 1.758-fold (Chen liver dataset [26], *P*=3.80e-13) and 2.215-fold (Wurmbach liver dataset [25], *P*=1.02e-05). However, the histopathological type of the other two datasets in XPO1 and one dataset in CSE1L was not HCC (Figure 1); thus, their results were not listed in Table 1. Next, the mRNA expression patterns of seven XPOs were measured by UALCAN, resources of which were based upon level 3 RNA-seq and clinical data from 31 cancer types of the TCGA database. As shown in Figure 2, significantly higher mRNA expression levels of all XPOs were found in primary HCC cancer tissues compared with normal liver tissues (*P*<0.05). Taken together, these results implied that the transcriptional expression of XPOs is up-regulated in HCC cancer tissues.

**Figure 1:** XPO gene expression in 20 different cancer types XPOs mRNA expression (cancer tissue vs. normal tissue) was analyzed using the ONCOMINE database. The numbers in colored cells show the quantities of datasets with statistically significant mRNA overexpression (red) or underexpression (blue) of target genes. Cell colors were determined by the best gene rank percentile for the analysis within cells. Analysis conditions required the following thresholds: gene rank percentile (10%), *P*-value (0.05) and fold change (1.5).

**Figure 2:** Transcription levels of XPOs in HCC cancer tissues and normal liver tissues Expression panels for XPO1 (**A**), CSE1L (**B**), XPOT (**C**), XPO4 (**D**), XPO5 (**E**), XPO6 (**F**), and XPO7 (**G**) comparing the data between 50 normal individuals and 371 HCC patients in the TCGA database. ***P<0.001.

**Table 1:** Significantly up-regulated expression in the transcription levels of XPOs between HCC and normal liver tissues (ONCOMINE database)

XPO	HCC vs. Normal	Fold change	*P*-value	*t* test	Datasets/References
XPO1	HCC	1.642	2.27e-09*	7.439	Roessler liver [24]
	HCC	1.683	9.79e-54*	17.772	Roessler liver 2 [24]
	HCC	1.782	2.65e-07*	7.72	Wurmbach liver [25]
CSE1L	HCC	2.209	2.02e-08*	7.087	Roessler liver
	HCC	2.188	2.77e-75*	23.12	Roessler liver 2
	HCC	1.914	2.16e-05*	4.613	Wurmbach liver
	HCC	-2.482	4.27e-06*	−6.763	Chen liver [26]
XPOT	HCC	2.445	8.41e-63*	19.922	Roessler liver 2
	HCC	1.763	4.01e-14*	8.11	Chen liver
	HCC	-2.122	4.32e-07*	−6.069	Mas liver [27]
XPO4	N/A	N/A	N/A	N/A	N/A
XPO5	HCC	1.758	3.80e-13*	7.735	Chen liver
	HCC	2.125	1.02e-05*	5.498	Wurmbach liver
XPO6	N/A	N/A	N/A	N/A	N/A
XPO7	N/A	N/A	N/A	N/A	N/A

Abbreviation: N/A, not available.

* *P*<0.05 was considered statistically significant.

### Correlation between XPO transcription with HCC clinicopathological parameters

We next analyzed the relationship between XPO mRNA transcription levels and the clinicopathological parameters of HCC patients by UALCAN. As shown in Figure 3, the mRNA expression levels of all seven XPO family members were remarkably correlated with the patients’ individual HCC clinical stage. The highest mRNA expression of an XPO was found at stage 3 instead of stage 4. The reason for this observation may be the small number of patients at stage 4 (only six patients). In addition, the mRNA expression of seven XPOs was significantly related to tumor pathological grade (Figure 4). The higher mRNA expression levels of XPOs tended to correlate with a more undifferentiated pathological grade. Noticeably, the mRNA expression levels of CSE1L and XPOT/6 were highest in tumor pathological grade 4 (Figure 4B,C,F), while the highest mRNA expression levels of XPO1/4/5/7 were found in grade 3 (Figure 4A,D,E,G). In short, these results suggested that the transcriptional levels of seven XPO members are significantly related to clinicopathological parameters in HCC patients.

**Figure 3:** Relationship between XPO mRNA expression and HCC clinical stage Expression panels for XPO1 (**A**), CSE1L (**B**), XPOT (**C**), XPO4 (**D**), XPO5 (**E**), XPO6 (**F**), and XPO7 (**G**) based on HCC cancer clinical stage comparing the data between 50 normal individuals and 371 HCC patients in the TCGA database. *P<0.05; **P<0.01; ***P<0.001.

**Figure 4:** Relationship between XPO mRNA expression and HCC pathological grade Expression panels for XPO1 (**A**), CSE1L (**B**), XPOT (**C**), XPO4 (**D**), XPO5 (**E**), XPO6 (**F**), and XPO7 (**G**) based on HCC tumor grade comparing the data between 50 normal individuals and 371 HCC patients in the TCGA database. Pathological grading: Grade 1, well-differentiated; grade 2, moderately differentiated; grade 3, poorly differentiated and grade 4: undifferentiated. *P<0.05; **P<0.01; ***P<0.001.

### Prognostic values of XPO mRNA levels in HCC

Furthermore, the open online tool GEPIA was used to analyze the prognostic values of XPOs in HCC patients. As shown in Figure 5, higher mRNA expression levels of XPO1 (*P*=0.0037), CSE1L (*P*=0.0067), XPOT (*P*=0.0079), XPO4 (*P*=0.0068), XPO5 (*P*=1.8e-05) and XPO6 (*P*=0.0024) predicted worse OS. However, XPO7 mRNA expression showed no significant association with OS (*P*=0.08, borderline significance). The results in Figure 6 showed that higher mRNA expression levels of XPO1 (*P*=0.047), CSE1L (*P*=0.0048), XPO5 (*P*=1.8e-7) and XPO6 (*P*=0.026) were associated with short DFS in HCC patients, but higher mRNA expression levels of XPOT (*P*=0.26), XPO4 (*P*=0.51) and XPO7 (*P*=0.052, borderline significance) were irrelevant to DFS. Thus, the mRNA expression levels of XPO1, CSE1L, XPOT, XPO4/5/6 are significantly associated with the prognosis of HCC patients.

**Figure 5:** OS difference based on XPO mRNA levels in HCC patients High XPO1, CSE1L, XPOT and XPO4/5/6 (**A–F**) mRNA expression levels were remarkably associated with poor OS in HCC patients, while that of XPO7 (**G**) was not (*P*=0.08, borderline significance).

**Figure 6:** DFS difference based on XPO mRNA levels in HCC patients High XPO1, CSE1L and XPO/5/6 (**A,B,E,F**) mRNA expression levels were associated with poor DFS in HCC patients, while those of XPOT/4 (**C,D**) were not and that of XPO7 (**G**) was uncertain (*P*=0.052, borderline significance).

### XPO genetic alterations and their association with HCC prognosis

To further explore the sequence mutations in XPO family members in HCC patients, the TCGA database and the c-BioPortal website were applied. As shown in Figure 7A, a high frequency of mutations was found in XPOs (44%, 158 of 360 HCC patients). The highest mutation rate was observed in XPO7 (46/360, 13%) compared with XPO1 (24/360, 7%), CSE1L (34/360, 9%), XPOT (28/360, 8%), XPO4 (28/360, 8%), XPO5 (24/360, 7%) and XPO6 (28/360, 8%). The main genetic alterations involved mRNA up-regulation in XPO1 (17/24, 70.8%), CSE1L (32/34, 94.1%), XPOT (25/28, 89.3%), XPO4 (23/28, 82.1%) and XPO6 (20/28, 71.4%), DNA amplification in XPO5 (21/24, 87.5%) and XPO6 (20/28, 71.4%) and DNA deletion in XPO7 (21/46, 45.65%). The Kaplan–Meier plot and log-rank test showed that HCC patients with XPO alterations had worse OS (Figure 7B, *P*=0.00271), but this situation was not the same for DFS (Figure 7C, *P*=0.0949). These results implied that sequence alterations in XPOs are related to the prognosis of patients with HCC.

**Figure 7:** XPO expression and mutation analysis in HCC (**A**) OncoPrint in c-BioPortal showed the distribution and proportion of samples with alterations in XPOs. (**B**) XPO alterations were associated with worse OS in HCC patients. (**C**) XPO alterations did not correlate with DFS in HCC patients.

### Network analysis of signaling pathways affected by XPO mutations in HCC

After analyzing the XPOs’ genetic alterations and their prognostic values in HCC patients, the 50 neighboring genes related to the XPO mutants were analyzed, and an integrated network was constructed on c-BioPortal. As expected, RAD21, NUP133, RRM2B, PPP2CB, YWHAZ and 45 other genes were significantly associated with XPO mutations (Figure 8A). The functions of the XPOs and their alteration-related genes were analyzed by GO, KEGG and DAVID. GO analysis mainly includes three aspects: biological process, cellular components and molecular functions. Regarding the biological process (Figure 8B), the results showed that GO:0006606 (protein import into the nucleus), GO:0006405 (RNA export from the nucleus), GO:0006611 (protein export from the nucleus), GO:0051301 (cell division) and GO:0000972 (transcription-dependent) were highly associated with XPO sequence alterations in HCC. For cellular components (Figure 8C), GO:0031080 (nuclear pore outer ring), GO:0031965 (nuclear membrane), GO:0000776 (kinetochore), GO:0005643 (nuclear pore) and GO:0034339 (nuclear periphery) were remarkably regulated by XPO alterations. For molecular function (Figure 8D), GO:0017056 (structural constituent of the nuclear pore), GO:0005049 (nuclear export signal receptor activity), GO:0005487 (nucleocytoplasmic transporter activity) and GO:0008536 (Ran GTPase binding) were also closely related to XPO alterations. KEGG analysis showed that cfa03013 (RNA transport), cfa04114 (oocyte meiosis), cfa04390 (hippo signaling pathway), cfa04110 (cell cycle) and cfa03015 (mRNA surveillance pathway) were influenced by XPO mutations in HCC (Figure 8E).

**Figure 8:** GO enrichment and KEGG pathway analyses of XPOs (**A**) Networks constructed in c-BioPortal showed the interaction relationship between XPO1, CSE1L and the 50 most frequently altered neighboring genes. GO functional enrichment analysis predicted three main functions of the target genes: (**B**) biological process, (**C**) cellular components and (**D**) molecular functions. (**E**) KEGG pathway analysis of XPO1, CSE1L and their 50 most frequently altered neighboring genes.

## Discussion

Currently, malignant tumors have been viewed as a set of diseases driven by the accumulation of genetic mutations and the disruption of epigenetic regulatory mechanisms [4,28]. Any alterations in XPO family members resulting from either genetic mutations or epigenetic changes could affect miRNA expression and consequently have profound effects on tumorigenesis [29,30]. Meanwhile, a growing body of studies have shown that the misregulation of nuclear export could result in various cancers [31–34]. Although some XPO family members have been confirmed to be related to HCC, their distinct roles remain to be elucidated. In the current study, the expression, mutations and prognostic values of XPOs in HCC were analyzed. We found that XPOs expression was up-regulated and correlated with tumor clinical stage, pathological grade and the prognosis of HCC. Moreover, frequent mutations in XPOs were observed and confirmed to be related to a worse prognosis in HCC.

XPO1 transports nearly 300 different cargo proteins across the nuclear envelope, including components in several key pathways that influence liver cancer growth and survival. For example, cancer cells utilize XPO1 to export p53, APC, p21, p27, Foxo, BRCA1, ATM and TopoI to the cytoplasm. Restriction of these key gatekeeper and caretaker proteins to the cytoplasmic compartment prevents them from suppressing tumor growth [35–37]. The overexpression of XPO1 has been found in various cancers, including liver, ovarian, pancreatic, gastric and lung carcinomas [13,38–41], and might serve as a potential prognostic indicator. In a human ovarian cancer study, it was found that the overexpression of XPO1 in the cytoplasm was prominently related to advanced tumor stage, poor differentiation and a higher mitotic rate, while higher XPO1 expression in the nucleus was associated with cyclooxygenase-2 expression and worse OS [42]. Similarly, Chen et al. [38] reported that XPO1 mRNA overexpression was correlated with decreased survival and platinum resistance in ovarian cancer. Thus, the inhibition of XPO1 is a promising therapeutic strategy for cancer treatment. KPT-330, a kind of selective inhibitor of nuclear export, could down-regulate XPO1 transcription and reduce the growth capability of HCC cells by increasing the expression of tumor suppressor proteins, such as p53 and p27, in the nucleus and reducing the concentration of oncogenes, such as c-Myc and c-Met [13]. Moreover, KPT-330 could cause the accumulation of p53 in the nucleus and the retention of p21 in the cytoplasm, which led to cell arrest and apoptosis in patients with gastric cancer [40]. Interestingly, KPT-330 can efficiently reverse anthracycline resistance by down-regulating XPO1 expression [43]. Azmi et al. [44] demonstrated that KPT-330 increased miR-145 expression in pancreatic ductal adenocarcinoma cells and inhibited tumor cell proliferation and migration capacities. Consistently, our analysis showed that XPO1 overexpression in HCC cancer tissues was correlated with poor pathological differentiation, advanced tumor clinical stage and a poor prognosis. Therapy targeting the XPO1 pathway might be a potential strategy to be explored.

CSE1L and its substrate, importin-α 1, were found to be up-regulated and significantly associated with a worse prognosis in HCC. Further mechanistic studies have indicated that X-linked inhibitor of apoptosis and p53 collaboratively mediate CSE1L mRNA expression [45,46]. Wellmann et al. [47] reported that strong expression of CSE1L was not only positively associated with the degree of inflammation in hepatitis but also a key regulator in tumorigenesis in HCC. Another study indicated that CSE1L could interact with the gene mutS homolog-6 and was also associated with a poor prognosis in osteosarcoma patients [48]. Moreover, protein phosphatase-1 could interact with CSE1L to control the cell cycle and the proliferation of cancer cells through CSE1L dephosphorylation in colon adenocarcinoma [49]. In this study, the results suggested that CSE1L was overexpressed in HCC tissues and correlated with a poor prognosis. Further studies on the mechanism by which CSE1L promotes HCC progression are needed.

Significant up-regulation of XPOT (also named XPOT) was found in liver and breast cancers [14,32]. High expression of XPOT in 95 liver cancer tissues predicted a worse prognosis. The knockdown of XPOT caused cell cycle arrest in G_0_/G_1_ phase by down-regulating cell cycle regulators, such as cyclin-dependent kinase-1 and cyclin A [14]. XPOT was also found to be increased and strongly related to worse OS in breast cancer [32]. Similar findings were found in studies regarding XPO4 [15,16,50]. Consistent with these results, our analyses from different datasets suggest that XPOT and XPO4 may serve as promising biomarkers for HCC prognosis.

Conflicting roles for XPO5 have been found in different kinds of human cancers. On one hand, the significant overexpression of XPO5 was found in breast, prostate and medullary thyroid carcinomas [32,51,52]. Excessive XPO5 overrode the inhibitory effect of canonical miRNA–mRNA regulation, which resulted in cellular protein instability, cellular proliferation and tumor development in prostate cancer [51]. Moreover, XPO5 was overexpressed in medullary thyroid carcinomas harboring RET mutations [52]. Consistent with these findings, our study showed that XPO5 overexpression was significantly related to HCC clinical stage, pathological grade and worse survival. On the other hand, decreased expression of XPO5 had been found in liver and bladder cancers [17,53].The aberrant expression of XPO5 significantly suppressed cell proliferation, colony formation, growth in soft agar and tumorigenicity in nude mice collectively demonstrating that XPO5 functions as a tumor suppressor in the progression of HCC [17]. The up-regulation of XPO5 could down-regulate the expression of microRNAs including miR-21, which suppresses p53 function, and subsequently inhibit the development of bladder tumors [53]. The discrepancy in the roles of XPO5 described above may be due to the different tumor types and study models.

XPO6 was overexpressed and associated with metastatic potential and a poor prognosis in prostate cancer tissue [54]. Consistent with these findings, our analysis revealed higher XPO6 mRNA expression in HCC cancerous tissues compared with paracancerous liver tissues, and it was significantly related to HCC clinical stage and pathological grade. XPO7 was recently reported to be down-regulated in both high-grade and low-grade differentiated tumors in epithelial ovarian carcinoma, and its low mRNA expression was associated with worse OS [55,56]. Interestingly, in the current study, significantly higher mRNA expression of XPO7 was found in HCC tissues and correlated with HCC clinical stage and pathological grade. Furthermore, we found that high XPO7 expression seemed to correlate with HCC prognosis (OS and DFS, borderline significance). Further experiments are needed to be performed to determine the exact role of XPO7 in HCC in the future.

Gene variants might modulate oxidative stress, iron metabolism, inflammatory and immune responses, DNA repair mechanisms and cell cycle regulation and consequently contribute to the tumorigenesis of HCC [57]. In the current study, the mutation frequency in XPO subunits was relatively high in HCC, and DNA sequence alterations mainly occurred in XPO7. In addition, the type of mutations may be associated with XPO mRNA expression levels. A previous study showed that DNA copy number amplifications could activate the mRNA expression levels of oncogenes [58]. More mRNA products could be found in genes with higher copy number variations and *vice versa* [59]. However, gene mutations are one of the many factors that affect transcriptional levels. Epigenetic changes, including DNA methylation, histone acetylation and methylation, noncoding RNAs, and post-translational modifications, are also main drivers involved in tumorigenesis independent of changes in the DNA sequence [60]. In the current analysis, we found that XPO mutations were related to mRNA up- or down-regulation, DNA amplification or deletion etc. These alterations were associated with OS in HCC patients. However, the potential molecular mechanism remains unclear and requires further investigation.

Therefore, we hypothesized that aberrant expression of XPOs may promote the proliferation and anti-apoptotic ability of HCC cells by enhancing the nuclear output of tumor suppressor factors (such as TP53) in the nucleus of HCC. On the other hand, we acknowledged that there were some limitations to our study. All data analyzed were retrieved from online databases. We did not perform further experiments on the potential mechanisms of XPOs in HCC. Together with other findings discussed above, our analyses suggested that XPOs play oncogenic roles in HCC. Future studies including immunohistochemistry and experiments on HCC cell lines or animal models could be used to investigate the detailed mechanism between XPOs and HCC.

## Conclusion

Our results showed that XPO family members were significantly overexpressed in HCC tissues, and their mRNA levels were significantly correlated with the clinical stage and tumor pathological differentiation grade. High mRNA expression of XPO1, CSE1L, XPOT and XPO4/5/6 significantly was correlated with OS, and high mRNA expression of XPO1, CSE1L and XPO5/6 was positively correlated with DFS. In addition, the mutation rate of XPO7 was the highest in HCC, and genetic changes in all XPOs examined were related to worse OS. These results suggest that XPOs might be potential biomarkers for predicting survival in HCC patients.

## Abbreviations

APC: Anaphase Promoting Complex or Cyclosome
ATM: Ataxia Telangiectasia Mutated
BRCA1: Breast Cancer Type1 Susceptibility Protein
DAVID: Database for Annotation, Visualization and Integrated Discovery
DFS: disease-free survival
Foxo: Forkhead Box O
GEPIA: Gene Expression Profiling Interactive Analysis
GO: Gene Ontology
HCC: hepatocellular carcinoma
HEAT: Huntingtin, Elogation factor 3, protein phosphatase 2A (pp2A) and the yeast kinase TOR1
KEGG: Kyoto Encyclopedia of Genes and Genomes
OS: overall survival
RET: Rearranged during Transfection
TCGA: The Cancer Genome Atlas
XPO: exportin
